# Research Progress of PCNA in Reproductive System Diseases

**DOI:** 10.1155/2021/2391917

**Published:** 2021-10-21

**Authors:** Jing Pan, Jianwei Zhang

**Affiliations:** ^1^The First Clinical College, Shandong University of Traditional Chinese Medicine, Jinan, Shandong, China; ^2^Hospital Affiliated to Shandong University of Traditional Chinese Medicine, Jinan, Shandong, China

## Abstract

Reproductive system diseases have become a public health problem that endangers human physical and mental health. The causes of reproductive diseases are complex and diverse. From a biological point of view, abnormal cell proliferation may affect important physiological functions of reproductive organs and cause various gynecological or andrological diseases. Proliferating cell nuclear antigen (PCNA) is the most commonly used indicator for detecting cell proliferation activity. The up- or downregulation of its expression is of great significance in reproductive system diseases. This review summarizes the significance of the latest research on PCNA expression in reproductive system diseases.

## 1. Introduction

Infertility is a medical problem affecting ten to fifteen percent of couples worldwide [1]. In recent years, the number of younger patients with infertility has increased. About 10% of couples of childbearing age in the United States have reproductive disorders, and this percentage is gradually increasing [2]. In the 21st century, infertility has become the third most common disease after tumors and cardiovascular and cerebrovascular diseases in China. Therefore, diseases of the reproductive system are an important factor that seriously endangers human physical and mental health [3]. Unfortunately, such diseases are commonly characterized by a lack of symptoms, and thus, a high proportion of patients do not see a physician. Furthermore, among those that do seek medical help, a high proportion undergoes unreasonable treatments, leading to various serious complications, including aggravating any infertility. This further reduces the level of reproductive health and directly affects the quality of life.

Proliferating cell nuclear antigen (PCNA) is an accessory protein of DNA polymerase *δ* with a unique ring structure. It is ubiquitous in proliferating eukaryotic cells and plays coordinating roles in the replication of deoxyribonucleotides, cell division, and proliferation [4]. PCNA is the most commonly used indicator for detecting tumor cell proliferation activity in recent years [5]. Most reproductive system diseases, including uterine fibroids (UFs), endometriosis (EM), adenomyosis (ADS), premature ovarian failure (POF), polycystic ovarian syndrome (PCOS), endometrial cancer (EC), cervical cancer (CC), ovarian cancer (OC), prostate cancer (PCa), and nonobstructive azoospermia (NOA), are caused by abnormal cell proliferation. This abnormal proliferation may be an important factor in determining the development or potential prognosis of various reproductive system diseases. Its regulatory function in the occurrence and development of reproductive system diseases is summarized in Figure 1.

As a function conversion factor, PCNA interacts with a variety of cytokines through different regulatory methods and participates in many important cellular events, such as chromatin remodeling, DNA damage repair, and apoptosis. To better understand the relationship between reproductive system diseases and PCNA and efficiently apply PCNA for early diagnosis, this review summarizes the importance of PCNA in a variety of abnormal proliferative diseases in the reproductive system and its involvement in related pathogenic processes.

## 2. Research on PCNA in Gynecology

The clinical causes of female infertility, including UFs, EM, ADS, POF, PCOS, EC, CC, and OC, are complex and numerous. These disorders may involve impairments at multiple points such as ovulation, sperm-egg recognition and fusion, and embryo implantation. Problems in these areas are often inseparable from abnormal cell proliferation, and the expression of PCNA is an important indicator of cell proliferation.

### 2.1. PCNA and UFs

UFs are the most common benign tumors in female reproductive organs. The most frequent and burdensome symptoms include severe uterine bleeding, pelvic pain, urinary incontinence, constipation, and, in patients of reproductive age, infertility or miscarriages [6, 7]. The risk of developing UFs increases with age. The growth of myomas involves an imbalance between cell proliferation and death. A selective progesterone receptor modulator, ulipristal acetate, is registered as a drug for the preoperative management of symptomatic myomas to reduce the size of tumors and eliminate abnormal uterine bleeding associated with fibroids [8–10]. It has been confirmed that PCNA expression decreases owing to the influence of ulipristal acetate [11]. Research results have also shown that ulipristal acetate reduces the volume of fibroids. This effect may be related to the decrease in PCNA and the increase in cell apoptosis in fibroids [12]. The elevated expression of PCNA in UFs may involve the increased levels of hypoxia-inducible factor-1*α*, AKT phosphorylation, vascular endothelial growth factor (VEGF), and collagen that promote microangiogenesis [13, 14]. Resveratrol, which is found in peanuts, grapes, and other plants, is a polyphenolic plant antioxidant with antiproliferative effects on several cancer cells, including breast and prostate cancers. It can significantly suppress fibroid growth in vivo and decrease the proportion of cells showing higher expression of PCNA [15]. This helps to decrease the volume and proliferation activity of uterine fibroids.

### 2.2. PCNA and EM

EM is a common gynecological disease in women. It is formed by active endometrial cells that are implanted outside the endometrium. Dysmenorrhea, chronic pelvic pain, menstrual abnormalities, and infertility are the main symptoms. Increased expression of PCNA is a known diagnostic marker for endometrial hyperplasia and EM. Montenegro et al. [16] used a rat model to evaluate the effect of physical exercise on EM and showed that the reduction in the size of EM lesions after exercise was related to the decrease in PCNA levels. It was verified that the PCNA level was positively correlated with the size of the endometriotic lesions. Women with EM have a lower body mass index and decreased body fat compared to those without the disease, and a gene expression analysis showed that microRNA (miRNA/miR)-Let-7b and miR-342-3p affected the expression of PCNA in the fat cells of women with EM [17].

Understanding the molecular and cellular causes of EM may provide new targets for treatment and restrict the systemic effects of the disease. Berberine (BBR), which is a typical component of *Coptis chinensis* Franch, is a potential treatment for endometrial cancer (EC) that inhibits the growth and metastasis of EC cells through the miRNA/miR-101/cyclooxygenase-2/prostaglandin E2 signaling pathway [18]. Gu and Zhou [19] demonstrated that 80 *μ*M BBR significantly suppressed the proliferation and colony formation of human endometrial stromal cells by downregulating the expression of miR-429 and inhibiting the expression of the PCNA protein, which provided a theoretical basis for using BBR to treat EM. Furthermore, some data suggest that RNA crosstalk is a crucial factor in the development of EM. Thus, PCNA may serve as an emerging target for the treatment of EM-related infertility in women of childbearing age [20].

### 2.3. PCNA and ADS

ADS is a diffuse or localized pathology in which the endometrial glands and stroma invade the myometrial wall. Similar to EM, it is a common estrogen-dependent uterine disorder and problematic disease in gynecology. ADS results in abnormal uterine bleeding, dysmenorrhea, and subfertility [21, 22]. The denomyotic junctional zone (JZ) plays an important role in ADS pathogenesis. JZ dysfunction has been suggested as a causative factor in the development of ADS [23]. Wang et al. [24] demonstrated that both PCNA mRNA and protein expression were significantly higher in the proliferative than the secretory phase of the menstrual cycle in normal JZ smooth muscle cells. However, the levels of these two indexes in patients with ADS were elevated, and the cyclic changes disappeared. Therefore, the combined application of these two indicators can improve the accuracy of diagnosis and prognosis assessment of patients with ADS. Furthermore, vimentin staining in adenomyotic epithelial cells is also increased, along with increased staining of VEGF and PCNA [25]. Upregulation of the expression of these proliferation and angiogenesis markers may indicate the pathogenesis of ADS.

### 2.4. PCNA and POF

Normal ovarian function is characterized by a short cell growth cycle and rapid proliferation that has some similarities with tumor cells; however, primitive ovarian follicle cells have no ability to regenerate. POF develops because of decreased oocyte storage, follicle arrest, or uncontrolled apoptosis. POF may also be caused by excessive activation of cell apoptosis during ovulation or a lack of healthy follicle development [26]. Wang et al. [27] used a POF mouse model to suggest that niacin may play an important role in the treatment of POF by increasing the level of PCNA, promoting the growth of follicles in immature oocytes, and reducing cell apoptosis. The results of that study may benefit women with POF or anovulatory diseases.

When treating some cancers with chemotherapy or radiotherapy, ovarian cell apoptosis or death is more serious due to DNA damage [28, 29]. This finding may provide clinical medication ideas to improve the ovarian function of cancer survivors. The chemotherapy process often causes significant toxicity in the reproductive system as it has deleterious effects on follicle formation, leading to irreversible POF. Cyclophosphamide (CP) has been widely used clinically to treat autoimmune diseases and ovarian cancer (OC). The side effects of CP as a chemotherapeutic alkylating agent include POF. Coenzyme Q10 (CoQ10) has a positive impact on the reproductive system due to its antioxidant properties, protecting cells from free-radical-mediated oxidative damage and apoptosis. A study has shown that the expression of PCNA and follicle-stimulating hormone receptor mRNA in CP-treated NMRI mice was reduced. In addition, the in vitro fertilization rate and embryo development were also affected, whereas the application of CoQ10 successfully reversed these changes [30]. The use of fenofibrate (FEN), alone or in combination with triptorelin, can improve the expression of PCNA [31]. The clinical application of FEN promoted the growth of follicles and protected the ovaries from the adverse effects induced by CP. Pretreatment with carvacrol or thymol significantly enhanced follicular development by improving the reduction in PCNA expression [32]. Niacin, CoQ10, FEN, triptorelin, and carvacrol can be considered effective protective therapies for the cytotoxic treatment of infertile women with POF, and PCNA may serve as a diagnostic and prognostic marker.

### 2.5. PCNA and PCOS

PCOS is an endocrine disorder. Apart from anovulation/oligoovulation and an abnormal androgen-to-estrogen ratio in serum, another characteristic and diagnostic criterion of PCOS is the presence of multiple cystic follicles in the ovary. The ovaries of women with PCOS show more cystic follicles that do not have the potential to develop into dominant follicles, leading to abnormal ovulation. The granular cell layer surrounding these follicles shows signs of atresia, degradation, and hypertrophy, indicating abnormal proliferation and/or apoptosis. Granular cells (GCs) are essential for providing oocytes with nutrients and growth regulators during oocyte development. The reduced expression of PCNA in cystic follicles is accompanied by downregulation of the cystic fibrosis transmembrane conductance regulator, which is required for normal follicle development and causes abnormal follicular development in PCOS [33]. GCs are the main source of VEGF production [34]. VEGF is one of the major regulators of angiogenesis and plays an important role in multiple diseases affecting the ovary, such as PCOS. A previous study demonstrated a decrease in PCNA protein levels in the luteinized GCs of women with PCOS. This may demonstrate that the downregulation of PCNA may disrupt the proliferation of GCs and cause the “arrest” of follicle growth, resulting in disordered folliculogenesis [35].

### 2.6. PCNA and EC

EC is the most frequent cancer in the female reproductive tract, with an increasing incidence rate, particularly among younger patients. Although most patients are diagnosed in the early stages of EC, some show poor prognosis and a high risk of recurrence and metastasis. Numerous studies have demonstrated an association between tumor progression and long noncoding RNA expression levels. For example, H19 is increased in various cancers, including EC [36]. Knockdown of H19 slowed tumor growth, promoted apoptosis, and upregulated miR-20b-5p expression, but lowered the expression of PCNA in vivo, thereby providing a novel target for diagnosing and treating EC [37]. P53, an important tumor suppressor, is dysregulated in numerous cancers [38–40]. Studies have shown that p53 is related to the progression and staging of EC and PCNA is the downstream regulatory target of p53. This indicates that the expression of PCNA is closely related to the prognosis and progression of EC [41]. Human epididymis protein 4, a secreted glycoprotein, is overexpressed in EC and modulates protein levels of the cell cycle marker, PCNA [42]. This may contribute to EC progression and/or metastasis. It has been reported that UFs have a protective effect on EC patients, and one meta-analysis identified that PCNA was overexpressed in a case of UFs and implicated as an EC inhibitor in the pathway analysis [43]. Geraniol exerts antitumor activity both in vitro and in vivo. Inhibition of PCNA expression by geraniol is a manifestation of its antiproliferative actions and protects against EC [44]. APOBEC1 complementation factor, an oncogene in many cancers, is highly expressed and closely related to the prognosis and progression of EC by downregulating the expression of PCNA [41].

### 2.7. PCNA and CC

CC is one of the most prevalent malignancies in women globally. A 50%–75% decrease in CC mortality (especially squamous CC) has occurred over the past 50 years, but the disease remains the third most common cancer in developing countries [45]. The DNA replication pathway has been suggested to have the strongest association with the prognosis of squamous CC, and PCNA was significantly correlated with survival [46]. The volatile anesthetic, isoflurane, activates the histone deacetylase 6 pathway, accompanied by the upregulation of PCNA protein expression, thereby promoting cervical carcinogenesis [47]. PCNA was significantly correlated with shorter overall survival in patients with CC [48]. Lv et al. [49] used CC as an example to conduct a systematic review and meta-analysis of the clinical effects of PCNA. The findings suggested that PCNA expression was significantly associated with poor 5-year survival, advanced stage, or higher World Health Organization grade, which indicated it might be a useful prognostic and diagnostic biomarker or an effective therapeutic target in CC or other cancers.

In vivo assays have shown that miR-326 can inhibit the expression of the PCNA protein, decrease the weight and slow down the growth of tumors, play a critical role in CC, and have potential as a biomarker or therapeutic target for CC [50]. Overexpression of peroxiredoxin 1 significantly promotes proliferation and inhibits apoptosis by increasing the expression of PCNA in human CC tissue and is closely related to tumor staging, lymphatic metastasis, and differentiation [51]. There have been results showing that the expression of PCNA in cervical intraepithelial neoplasia tissue and cervical squamous cell carcinoma is significantly higher than that in normal cervical epithelium tissue. In addition, the upregulation of PCNA expression is related to the degree of differentiation, International Federation of Obstetrics and Gynecology grade, lymph node metastasis, depth of cancer invasion, and human papilloma virus infection [52]. PCNA is highly expressed in squamous CC and is related to malignant tumors.

To provide targeted treatment for cancer patients and improve their quality of life, there is an urgent need to explore the underlying molecular mechanisms of CC cell proliferation and metastasis. High levels of four-and-a-half LIM domains protein 2 and PCNA are related to the occurrence, aggravation, and poor prognosis of CC [53]. Overexpression of the receptor for advanced glycation end products promotes the proliferation of squamous CC cells and increased PCNA expression [54]. The epigenetic regulator, G9a, is involved in cancer invasion and metastasis and suppresses xenograft tumor growth in a mouse model. These effects are linked to a decrease in microvessel density and PCNA expression [55]. Studies have shown that the overexpression of RIZ1, a tumor suppressor gene, combined with radiotherapy, increases DNA damage and facilitates apoptosis in CC cells by reducing the expression of PCNA [56]. These current findings provide novel insights into the pathophysiology of CC and may have important value for designing targeted therapy.

### 2.8. PCNA and OC

OC is a common tumor of the female genital organs, with an incidence rate similar to those of CC and EC, as well as the highest death rate among malignant gynecological tumors [57, 58]. Due to the atypical or asymptomatic nature of the early stage of OC, most patients diagnosed with this disease are already in the late stage, and OC has become the fifth primary cause of death among women [59]. Researchers using the immunohistochemical SP method found that the expression level of PCNA in OC tissues was significantly higher than that in benign ovarian tumor tissues and normal ovarian tissues and confirmed that the levels of CD24, B7-H4, and PCNA in OC tissues were positively correlated with each other [60]. These three indicators are closely related to the occurrence, development, invasion, and metastasis of OC, and their combined detection has clinical significance for the early diagnosis of OC and the screening of high-risk patients. One study explored distal-less homeobox 6 antisense 1 as an oncogene in OC and found that it accelerated tumor progression by upregulating four-and-a-half LIM domains protein 2 and PCNA via miR-195-5p. This provides new theoretical support for the targeted therapy of OC [61].

High-purity Baiye no. 1 tea flower saponin can effectively inhibit the proliferation of OC cells in a concentration-dependent manner as evidenced by the inhibition of cell viability, reduction in colony forming ability, and suppression of PCNA protein expression [62]. This study demonstrates that Baiye no. 1 tea flower saponin has the potential to be used as a nutraceutical for the prevention and treatment of OC.

Nuclear insulin-like growth factor-1 receptor, which is related to poor prognosis of cancer, increases DNA damage tolerance in serous OC [63]. The downregulation of bone morphogenetic protein endothelial cell precursor-derived regulator decreased the expression of PCNA, which was related to a decrease in ovarian epithelial malignant tumors and a higher survival rate [64]. Cotreatment with protein kinase G II and L-arginine inhibited the expression of PCNA in OC cells and was speculated to be a cancer inhibitor with a wide range of effects [65]. Overall, different anticancer drugs and multipathway studies have shown that a decrease in OC cell growth is closely related to the decrease in PCNA expression. This is of far-reaching significance for exploring the underlying disease mechanism and designing targeted therapy.

## 3. Research on PCNA in Andrology

The World Health Organization estimates that 9% of couples worldwide struggle with fertility issues, and approximately half of all cases are caused by male infertility [66]. Leydig cells are one of the main cell types in the testis and the primary site for androgen synthesis and secretion. Leydig cells are distributed in clusters between the seminiferous tubules and can promote the development of reproductive organs and spermatogenesis in males. Additionally, oxidative stress and apoptosis in Leydig cells are closely related to testicular function [67, 68]. Studies have found that 2,2′,4,4′-tetrabromodiphenyl ether upregulates the expression of PCNA in the testis and induces the proliferation of Leydig cells [69]. This has very important clinical significance for the treatment of male infertility.

### 3.1. PCNA and PCa

According to cancer statistics, prostate cancer is one of the most commonly diagnosed cancers in men [70] and is the second leading cause of cancer-related mortality among American men [71]. In South Korea, the incidence of prostate cancer has also increased significantly due to an increase in average life expectancy, Westernized eating habits, and increased awareness of prostate cancer screening [72]. In China, the incidence of prostate cancer is increasing year by year, and the disease significantly affects the quality of life and life expectancy of men over 60 years of age. The expression of PCNA is directly and negatively regulated by mesenchymal stem cell-derived exosomes that contain miR-143, which inhibit the proliferation, migration, and invasion of prostate cancer cells and promote apoptosis, thus hindering tumor growth [73].

### 3.2. PCNA and NOA

NOA is defined as the absence of spermatozoa in semen due to impaired spermatogenesis. Among men referred for an andrological diagnostic work-up, azoospermia is observed in 10%–15% of cases, with the majority of patients suffering from NOA [74]. In contrast to the treatable form of hypogonadotropic hypogonadism, primary testicular failure that causes NOA is the most serious form of male factor infertility [75]. At the histological level, the patterns of testicular damage range from hypospermatogenesis and spermatogenic arrest to Sertoli cell-only syndrome [76]. Sufficient sperm depends on the proliferative activity of spermatogonia and the loss of germ cells during meiosis and spermatogenesis. PCNA is a nuclear matrix protein involved in DNA synthesis and repair during spermatogenesis. PCNA is also a useful marker for diagnosing germinal arrest, which is the result of deterioration in DNA synthesis [77]. In one study, clomiphene citrate was used to treat infertile men with NOA; subsequent testicular sperm extraction showed that most tubules (>70%) exhibited no tubular lumen or regular seminiferous epithelium, but there were a large number of spermatogonia-like cells that exhibited normally differentiated spermatogonia with enhanced proliferation activity (positive for PCNA) [78]. The mechanism for effective spermatogenesis involves germ cell type-specific posttranslational modifications of histones, and histone variants play an important role. There is a significant positive correlation between histone H3.5, which is expressed specifically in spermatogonia and primary spermatocytes [79], and PCNA expression [80]. This information provides a diagnosis and treatment strategy for male infertility.

## 4. Conclusions and Future Directions

PCNA was initially identified as an essential factor for cell proliferation. It has been widely reported that the overexpression of PCNA is found in various gynecological disorders, including UFs, EM, ADS, POF, PCOS, EC, CC, and OC. Therefore, PCNA is suggested as a useful prognostic and diagnostic biomarker for the abovementioned diseases and as a therapeutic target to inhibit cell proliferation. However, considering the molecular progression of the abovementioned cancers and clinically confirmed treatments, it is more likely that a combinatorial application of PCNA with some transcription regulators, coregulators, and enzymes, such as nuclear insulin-like growth factor-1 receptor, bone morphogenetic protein endothelial cell precursor-derived regulator, CD24, B7-H4, histone deacetylases, peroxiredoxin 1, P21, and P53, will be effective for the diagnosis of gynecological cancers at different stages. Furthermore, these molecules, but not PCNA alone, are also potential therapeutic targets for better clinical strategies, and the targeted application of antibodies against the abovementioned molecules may provide better clinical results for women with infertility. In addition, further investigation of existing clinical applications of specific treatments for gynecological disorders, such as *C. chinensis* for EM and geraniol for EC, may reveal specific theories and strategies for treating specific gynecological diseases. The same strategies may also be applied for prostate cancer, but not another common andrological disorder, NOA, which is caused by the impairment of spermatogenesis and needs a way to enhance PCNA activity in spermatogonia. Few clinical cases are included in this review, and multicenter, large-sample clinical research is still needed. In addition, the various pathways and approaches can be explored in depth and comprehensively from theoretical and animal experiments. Finally, multimolecule and multiomics crossover research can be conducted.

## Figures and Tables

**Figure 1:** PCNA expression regulation of proliferative genes in the occurrence and development of gynecological and andrological diseases.

## Data Availability

The data used to support the findings of this study are available from the corresponding author upon request.
